The article "Anti-α-synuclein immunotherapy reduces α-synuclein propagation in the axon and degeneration in a combined viral vector and transgenic model of synucleinopathy" was retracted in 2026. Reasons: duplicated images; overlap with earlier publications; unreliable data.

# Anti-α-synuclein immunotherapy reduces α-synuclein propagation in the axon and degeneration in a combined viral vector and transgenic model of synucleinopathy

**DOI:** 10.1186/s40478-016-0410-8

**Published:** 2017-01-13

**Authors:** Brian Spencer, Elvira Valera, Edward Rockenstein, Cassia Overk, Michael Mante, Anthony Adame, Wagner Zago, Peter Seubert, Robin Barbour, Dale Schenk, Dora Games, Robert A. Rissman, Eliezer Masliah

**Affiliations:** 1 Departments of Neurosciences, University of California, La Jolla, San Diego, CA 92093 USA; 2 Prothena Biosciences Inc, 650 Gateway Boulevard, South San Francisco, CA 94080 USA; 3 Pathology, University of California, La Jolla, San Diego, CA 92093 USA; 4 Veterans Affairs San Diego Healthcare System, San Diego, CA 92161 USA; 5 University of California, 9500 Gilman Drive, La Jolla, San Diego, CA 92093-0624 USA

**Keywords:** α-synuclein, Animal model, Axonal transport, Immunization, Synucleinopathy

## Abstract

Neurodegenerative disorders such as Parkinson’s Disease (PD), PD dementia (PDD) and Dementia with Lewy bodies (DLB) are characterized by progressive accumulation of α-synuclein (α-syn) in neurons. Recent studies have proposed that neuron-to-neuron propagation of α-syn plays a role in the pathogenesis of these disorders. We have previously shown that antibodies against the C-terminus of α-syn reduce the intra-neuronal accumulation of α-syn and related deficits in transgenic models of synucleinopathy, probably by abrogating the axonal transport and accumulation of α-syn in in vivo models. Here, we assessed the effect of passive immunization against α-syn in a new mouse model of axonal transport and accumulation of α-syn. For these purpose, non-transgenic, α-syn knock-out and mThy1-α-syn tg (line 61) mice received unilateral intra-cerebral injections with a lentiviral (LV)-α-syn vector construct followed by systemic administration of the monoclonal antibody 1H7 (recognizes amino acids 91-99) or control IgG for 3 months. Cerebral α-syn accumulation and axonopathy was assessed by immunohistochemistry and effects on behavior were assessed by Morris water maze. Unilateral LV-α-syn injection resulted in axonal propagation of α-syn in the contra-lateral site with subsequent behavioral deficits and axonal degeneration. Passive immunization with 1H7 antibody reduced the axonal accumulation of α-syn in the contra-lateral side and ameliorated the behavioral deficits. Together this study supports the notion that immunotherapy might improve the deficits in models of synucleinopathy by reducing the axonal propagation and accumulation of α-syn. This represents a potential new mode of action through which α-syn immunization might work.

The article "Anti-α-synuclein immunotherapy reduces α-synuclein propagation in the axon and degeneration in a combined viral vector and transgenic model of synucleinopathy" was retracted in 2026. Reasons: duplicated images; overlap with earlier publications; unreliable data.

## Introduction

Synucleinopathies affect over 1 million people in the US alone [49]. This heterogeneous group of disorders includes idiopathic Parkinson’s disease (PD), PD dementia (PDD) and dementia with Lewy bodies (DLB) [48]. Synucleinopathies are clinically characterized by cognitive decline, behavioral alterations with hallucinations and depression, REM sleep behavior disorder, olfactory deficits, bowel movement alterations and dysautonomia [59]. The definitive diagnosis of synucleinopathies is made pathologically by the detection of Lewy bodies and neurites, which are composed mainly of α-synuclein (α-syn) and are found in neocortical, limbic and subcortical regions as well as in peripheral organs. In synucleinopathies, α-syn accumulates in synaptic terminals [5, 28, 58] axons [15, 18] and the neuronal cell body cytoplasm [61]. In these sites, α-syn accumulates as aggregated species (oligomers, protofibrils and fibrils) [9, 21, 25, 29, 30, 51, 63, 67, 68, 73]. Aggregated α-syn species are believed to cause neurodegeneration and to be transmitted from neuron to neuron via a prion-like propagation [32, 53].

Various neuropathological studies suggest that the spatial and temporal patterns of distribution of α-syn pathology in the CNS among the different types of synucleinopathies follow known patterns of synaptic connectivity [6, 14, 65]. This, in combination with recent studies showing that α-syn oligomers can be released by neurons and promote neurodegeneration and inflammation by propagating to other neurons [8, 12, 20, 37, 50] and glial cells [35], has strengthened the concept that cell-to-cell transmission of pathogenic forms of α-syn might play a role in the pathogenesis of synucleinopathies. Several mechanisms have been proposed to explain the cell-to-cell transmission of α-syn including prion-like seeding mediated by fibrils [37, 52, 53], release into the Interstitial fluid [27] or in micro-vesicles containing α-syn aggregates [10, 15, 26, 36], transmission via nanotubules [69] and trans-synaptic dissemination [7, 11, 22, 62]. Supporting the later hypothesis, recent studies have shown that injections of α-syn with viral vectors into the nucleus of vagus [22] or fibrils into the olfactory bulb [38, 47, 55, 56], striatum or limbic system [38] results in α-syn distribution along axons and synapses following known patterns of synaptic connectivity.

We have previously shown that active immunization against α-syn protects against neurodegeneration and reduces α-syn accumulation by promoting its degradation via lysosomal pathways [43] and reduces inflammation via fractalkine [39]. Likewise, passive immunization with antibodies against α-syn reduces memory and neurodegenerative deficits by promoting clearance of α-syn via autophagy [44] or microglia-dependent degradation [3]. Furthermore, immunization to certain epitopes of α-syn might also reduce α-syn propagation to glial and neuronal cells [3, 72], by blocking the C-terminal (CT) truncation of α-syn [19, 72] and prion-like propagation [66]. Moreover, we have recently shown that monoclonal antibodies against the proximal (1H7, aa 91-99) or distal C-terminus of α-syn (9E4 or 5C1, aa 118-126) reduced the cell-to-cell propagation of α-syn in an *in vitro* chamber system where acceptor and donor cells were separated by a membrane [19]. However, it is unclear if immunization might also abrogate the axonal transport and accumulation of α-syn in *in vivo* models of synucleinopathy. Therefore, we directly explored the effect of passive immunization against α-syn with the 1H7 antibody in a new mouse model of axonal transport and accumulation of α-syn. To model the axonal transport and accumulation of α-syn in vivo, a lentivirus containing the human α-syn was unilaterally delivered in the hippocampus by stereotaxic injection and α-syn protein was monitored on the ipsilateral and contra-lateral side, the later in both axonal projections (commissural fibers) and intraneuronal (neuronal transmission). The 1H7 monoclonal was selected because this antibody recognizes aggregated α-syn, reduces α-syn accumulation in the mThy1-α-syn transgenic (tg) mouse and has been shown to reduce the propagation in an *in vitro* cell based model [19]. Non-transgenic (non-tg), α-syn knock-out (KO) and mThy1-α-syn tg (line 61) mice received intra-cerebral injections with a lentiviral (LV)-human-α-syn vector construct followed by systemic administration of the monoclonal antibody 1H7 or isotype control IgG for 3 months. Passive immunization with 1H7 antibody reduced α-syn axonal transport and accumulation in the contra-lateral side and axonal degeneration and ameliorated the behavioral deficits, further supporting the notion that immunization against α-syn might be of therapeutic value for synucleinopathies.

The article "Anti-α-synuclein immunotherapy reduces α-synuclein propagation in the axon and degeneration in a combined viral vector and transgenic model of synucleinopathy" was retracted in 2026. Reasons: duplicated images; overlap with earlier publications; unreliable data.

## Materials and methods

### Mouse model of α-syn axonal transmission to the contralateral side and passive immunization

In this study we used groups of 3-4 month old female non-tg mouse littermates, homozygous α-syn KO and mice over-expressing human wt α-syn under the mThy1 promoter (mThy1-α-syn, Line 61) [57]. The wtα-syn tg mouse model was selected because these mice develop behavioral motor deficits [16], axonal pathology and accumulation of CT-cleaved α-syn and aggregates in cortical and subcortical regions [18] mimicking synucleinopathies [46]. The α-syn KO mice were obtained from Jackson laboratories (ID:003692, Maine, USA; B6;129X1-*Snca* ^*tm1Rosl*^/J) these mice were generated by replacing exons 3-7 with a PGK-neo cassette [1].

To characterize the model, groups of non-tg, α-syn-KO and α-syn tg mice received a single unilateral injections into the hippocampus of either LV-control (empty vector) or the LV-human-α-syn [4] (*n* = 10 per group) (2 μl at titer 2 x 10^9^ TDU). Mice were sacrificed for analysis 4 weeks after the injection. Lentivirus vectors were prepared by transient transfection of the three packaging plasmids and the vector plasmid in 293 T cells as previously described [60, 64]. Briefly, as previously described [40], mice were placed under anesthesia on a Koft stereotaxic apparatus and coordinates (hippocampus: AP 2.0 mm, lateral 1.5 mm, depth 1.3 mm) were determined as per the Franklin and Paxinos atlas [17]. The lentiviral vectors were delivered using a Hamilton syringe connected to a hydraulic system to inject the solution at a rate of 1 μl every 2 min. To allow diffusion of the solution into the brain tissue, the needle was left for an additional 5 min after the completion of the injection. Upon sacrifice, the brain was removed. In a subset of mice (*n* = 5 per group) the brains were post-fixed in phosphate-buffered 4% paraformaldehyde (pH 7.4) at 4 °C for 48 h for neuropathological analysis, while in the other subset (*n* = 5 per group) the brains were divided along the sagittal plane, snap-frozen, and stored at -70 °C for subsequent DNA analysis.

For the immunotherapy experiments, 19 non-tg, 17 α-syn KO and 16 α-syn tg mice were included in this randomized and double-blind study. Starting the day after lentivirus (LV) injection, mice were immunized with weekly intraperitoneal injections of 30 mg/kg of 1H7 (anti–α-syn 91-99) or 27-1 (control immunoglobulin G1 [IgG1]) for a period of 3 months (Fig. 1a). The 1H7 monoclonal antibody was generated with recombinant α-syn and has been shown to recognize with high affinity aggregated α-syn, to reduce α-syn accumulation, to protect against behavior deficits in the mThy1-α-syn tg and to block propagation in an *in vitro* cell based model [19]. Each cohort of non-tg, α-syn KO and α-syn tg mice received either the 1H7 antibody or the control mAb 27-1 as follows: α-Syn KO mice + 27-1 (control) *n* = 8; α-syn KO + 1H7 antibody *n* = 9; non-tg mice + 27-1 (control) *n* = 10; non-tg mice + 1H7 antibody *n* = 9; α-syn tg mice + 27-1 (control) *n* = 8; α-syn tg mice + 1H7 antibody *n* = 8. As a control, an additional group of *n* = 9 non-tg mice were injected with LV-control and treated with 27-1. To verify that the antibody permeated into the CNS, a subset of *n* = 6 α-Syn KO; *n* = 6 non-tg and *n* = 6 α-syn tg mice were injected in the tail vein with Alexa tagged 27-1 control mAb (*n* = 3 per group; 10 mg/kg) or 1H7 antibody (*n* = 3 per group; 10 mg/kg) prepared as previously described [44].

The article "Anti-α-synuclein immunotherapy reduces α-synuclein propagation in the axon and degeneration in a combined viral vector and transgenic model of synucleinopathy" was retracted in 2026. Reasons: duplicated images; overlap with earlier publications; unreliable data.

**Fig. 1:** Schematic overview of the experimental paradigm. **a** Study Design. α-Syn KO, non-tg, and α-syn tg mice were injected with LV-α-syn 1 week before beginning passive immunization with systemic (intraperitoneal) injections of either control IgG (27-1) or α-syn 91-99 antibody (1H7). Immunization occurred once a week for a total of 13 weeks. Water maze testing occurred 14 weeks after LV-α-syn injection. Mice were euthanized 16 weeks after LV-α-syn injection. **b** Schematic representation of the unilateral injection of LV-α-syn into the hippocampus. **c** Schematic representation of the α-syn molecule and the binding epitope of the 1H7 antibody. Area in red represents the central hydrophobic region [23, 24, 70]

Behavioral tests were performed at the end of the immunization protocol. Upon sacrifice, the whole brain was removed and post-fixed in phosphate-buffered 4% paraformaldehyde (pH 7.4) at 4 °C for 48 h for neuropathological analysis. All experiments were approved by the institutional animal use and care committee of the UC San Diego (UCSD) and were performed according to NIH guidelines for animal use.

### Behavioral testing

In patients with synucleinopathies, α-syn accumulates in cortical regions and the limbic system resulting in cognitive deficits [13]. In the mThy1-α-syn tg mice, CT-truncated and oligomeric α-syn accumulates in synapses and axons in the temporal cortex and hippocampus [18]. To evaluate spatial learning and memory, the Morris water maze was used as previously described [44]. Briefly, a pool (diameter 180 cm) was filled with opaque water (24 °C) and mice were first trained to locate a visible platform (days 1-3) and then a submerged hidden platform (days 4-7) in three daily trials, 2-3 min apart. Mice that failed to find the hidden platform within 90 s were placed on it for 30 s. The same platform location was used for all sessions and all mice. The starting point at which each mouse was placed into the water was changed randomly between two alternative entry points located at a similar distance from the platform. In addition, on the final day of testing, the platform was removed and the time spent by mice in the correct quadrant was measured (probe test). Time to reach the platform (escape latency) was recorded with a Noldus Instruments EthoVision video tracking system (San Diego Instruments, San Diego, CA), set to analyze two samples per second.

### PCR analysis of lentivirus expression

In addition to the cohort of mice used for behavior, DNA was extracted from the hippocampus, both ipsi- and contralateral to the site of the lentiviral injection with either LV-α-syn or LV-GFP, from a separate cohort of non-tg, α-syn KO and α-syn tg mice (*n* = 5), and PCR was performed to analyze the levels of virus. Total DNA was isolated from mice brains with the DNeasy Blood & Tissue kit (Qiagen). Real-time PCR analysis was performed using the StepOnePlus real-time PCR system (Applied Biosystems) with primers specific for the virus human α-syn (5’-TGT TGG AGG AGC AGT GGT GA-3’ and 5’-TGC CCA ACT GGT CCT TTT TG-3’) or GFP (5'- GGA GCG CAC GAT CTT CTT CA-3' and 5'-AGG GTG TCG CCC TCG AA-3’). Viral presence was calculated by the comparative threshold cycle (Ct) method using a standard curve of purified LV-α-syn and analysis of GADPH was performed as internal control.

The article "Anti-α-synuclein immunotherapy reduces α-synuclein propagation in the axon and degeneration in a combined viral vector and transgenic model of synucleinopathy" was retracted in 2026. Reasons: duplicated images; overlap with earlier publications; unreliable data.

### Immunohistochemical and neuropathological analysis

Analysis of α-syn accumulation was performed using free-floating coronal brain sections (40 μm). Brain sections were incubated overnight at 4 °C with a polyclonal antibody against total α-syn (1:500, affinity-purified rabbit polyclonal, Millipore) [45], an antibody against CT-truncated α-syn (SYN105) [18], or isotype controls (background levels), followed by incubations with secondary antibodies biotinylated (1:100, Vector Laboratories, Inc., Burlingame, CA), Avidin D-HRP (1:200, ABC Elite, Vector) and detection with 3,3’-diaminobenzidine [44]. All sections were processed simultaneously under the same conditions and experiments were performed in triplicate in order to assess the reproducibility of results.

Sections were analyzed with an Olympus BX41 digital video microscope equipped with a Optronics magna fire SP camera, LucisTM DHP unique contrast enhancement software and Image Pro ExpressTM for live image acquisition and processing at 630X magnification. For each section 4 areas of interest (1024 x 1024 pixels) within the hippocampal neuropil, CA1 region and axons above the hippocampus in the area ipsilateral and contralateral were analyzed in real time using the Image Pro Plus (Media Cybernetics) software. α-Syn levels of immunoreactivity in the hippocampus neuropil and in axons in the white matter tracts were expressed as corrected optical density (arbitrary units). Analysis was performed around the area of injection within a 50 μm ratio.

### Double immunolabeling and confocal microscopy

To evaluate the effects of immunization on the LV-α-syn driven axonal pathology and propagation, sections were immunolabeled with an antibody against the neurofilament marker SMI312 (1:100) [42, 60]. In addition, sections were double-immunolabeled with the CT- truncated-α-syn antibody SYN105 (1:500) [18] and the anti-human α-syn antibody SYN211 (Millipore). α-Syn propagation in the dystrophic axons was detected with the Tyramide Signal Amplification™-Direct (Red) system (1:100, NEN Life Sciences, Boston, MA), while the SYN211 was detected with a FITC-tagged antibody (Vector, 1:75). To evaluate the clearance of α-syn by microglia, briefly as previously described [33, 34] sections were double labeled with antibodies against α-syn (Millipore, 1:500) detected with Tyramide Signal Amplification™-Direct (Red) system and Iba-1 (a microglial marker, 1:2500, Wako) detected with FITC. All sections were processed simultaneously under the same conditions and experiments were performed in triplicate in order to assess the reproducibility of results. Sections were imaged with a Zeiss 63X (N.A. 1.4) objective on an Axiovert 35 microscope (Zeiss) with an attached MRC1024 LSCM (laser scanning confocal microscope) system (BioRad) [45]. Image analysis using Image J was utilized as previously described [41] to determine the percent of microglia displaying α-syn immunoreactivity.

The article "Anti-α-synuclein immunotherapy reduces α-synuclein propagation in the axon and degeneration in a combined viral vector and transgenic model of synucleinopathy" was retracted in 2026. Reasons: duplicated images; overlap with earlier publications; unreliable data.

### Statistical analysis

All experiments were done blind-coded and in triplicate. Values in the figures are expressed as means ± SEM. To determine the statistical significance, values were compared using Student’s t-test, one-way analysis of variance (ANOVA) with Dunnett’s post-hoc test or Tukey-Kramer post-hoc test, as indicated in each figure legend. The differences were considered significant if *p* values were less than 0.05.

## Results

### α-Syn transmits and accumulates in axons in the contralateral side following unilateral LV-α-syn injection into the hippocampus

To evaluate if antibodies against α-syn can reduce axonal transport and accumulation of α-syn in the contralateral side, we first developed a new animal model of neuronal α-syn transmission utilizing unilateral intra-hippocampal injections of LV-control or LV-α-syn into α-syn-KO, non-tg and α-syn tg mice (Fig. 1). Four weeks post LV-α-syn injection, brains were fixed and sectioned in the coronal plane and analyzed histologically. As expected, the α-syn-KO mice (Fig. 2a, b) did not show α-syn immunoreactivity, while non-tg mice (Fig. 2c, d), and α-syn tg mice (Fig. 2e, f) injected with the LV-control (empty vector) only showed punctate α-syn immunoreactivity restricted mostly to synaptic sites in both the ipsilateral or contralateral sides. In contrast, the α-syn KO mice injected with LV-α-syn showed intense α-syn immunoreactivity throughout the hippocampus in the ipsilateral site, including neuronal cell bodies and neuropil (Fig. 2g, h -- right panels). The trans-hippocampal axons (commissural fibers) and corpus callosum axons also displayed α-syn immunoreactivity. In the contralateral hippocampi, somatic α-syn immunoreactivity was detected in the molecular layer of the dentate gyrus and subiculum as well as in axons in the subiculum and corpus callosum (Fig. 2g, h -- left panels). The contralateral side displayed somatic α-syn aggregates ranging in size between 3-6 μm in diameter (Fig. 2g, h) and some of these structures appeared to be associated with dystrophic neurites (Fig. 2g, h).

The article "Anti-α-synuclein immunotherapy reduces α-synuclein propagation in the axon and degeneration in a combined viral vector and transgenic model of synucleinopathy" was retracted in 2026. Reasons: duplicated images; overlap with earlier publications; unreliable data.

**Fig. 2:** Immunohistochemical analysis of LV-αsyn in α-syn KO, non-tg, and α-syn tg mice. α-syn KO, non-tg and α-syn tg mice were evaluated 16 weeks after unilateral LV injection into the hippocampus. Total α-syn antibody was used for these experiments. **a** Representative low and (**b**) high magnification of LV-control injected ipsi-laterally in α-syn KO mice revealed complete absence of any α-syn immunoreactivity in the hippocampus. **c** Representative low magnification and (**d**) high magnification of α-syn immunoreactivity in the ipsi-lateral and contra-lateral sides following LV-control injection in non-tg mice. **e** Representative low and (**f**) high magnification of α-syn immunoreactivity in the ipsi-lateral and contra-lateral sides following LV-control injection in α-syn tg mice. **g** Representative low magnification and (**h**) high magnification of α-syn immunoreactivity in the ipsi-lateral and contra-lateral sides following unilateral LV-α-syn injection in α-syn KO mice. **i** Representative low magnification and (**j**) high magnification of α-syn immunoreactivity in the ipsi-lateral and contra-lateral sides following LV-α-syn injection in non-tg mice. **k** Representative low and (**l**) high magnification of α-syn immunoreactivity in the ipsi-lateral and contra-lateral sides following LV-α-syn injection in α-syn tg mice. Low magnification scale bar = 250 μm; high magnification scale bar = 25 μm. *N* = 5 per group

Non-tg mice (Fig. 2i, j) and α-syn tg mice (Fig. 2k, l) showed similar distributions of α-syn-KO, but with relative higher levels of pathology likely related to the baseline levels of α-syn expression. In both models, stronger immunoreactivity was detected in the ipsilateral hippocampus, as expected from the protein overexpression, including labeling of neurons and axons. In the contralateral hippocampi α-syn immunostaining was found in axons along the trans-hippocampal tracts (commissural pathway) and in dystrophic neurites (Fig. 2i-l, left panels). Since α-syn KO, non-tg, and α-syn tg mice injected with the LV-control (empty vector) did not show detectable increases in α-syn immunoreactivity in the ipsilateral or contralateral sides when compared to non-injected controls (Fig. 2a, f), all ensuing experiments focused on alterations in α-syn KO, non-tg, and α-syn tg mice injected with LV-α-syn.

The article "Anti-α-synuclein immunotherapy reduces α-synuclein propagation in the axon and degeneration in a combined viral vector and transgenic model of synucleinopathy" was retracted in 2026. Reasons: duplicated images; overlap with earlier publications; unreliable data.

To further confirm the neuritic localization of α-syn in the contralateral side of the α-syn KO mice, double immunolabeling was performed with antibodies (Ab) against α-syn and phosphorylated neurofilaments (p-NF, SMI312 Ab; axonal marker). Image analysis by confocal microscopy of the α-syn KO, non-tg, and α-syn tg mice indicated that about 40% of the α-syn aggregates along the hippocampus (Fig. 3a) and corpus callosum (Fig. 3b) in the contra-lateral side co-localized with the SMI312 antibody, indicating their intra-axonal locality, while the remainder surrounded the axons (Fig. 3b). To verify that the α-syn signal detected in the contralateral side was the results of the axonal transport and accumulation of the protein and not due to migration of the injected virus, PCR analysis for the viral human α-syn or GFP DNA was performed. First, to confirm that α-syn protein was migrating axonally rather than the virus, immunofluorescence analysis was performed of brain sections from mice injected with LV-α-syn. This study showed that granular and pyramidal cells in the ipsilateral side displayed strong α-syn immunostaining that extended to the neuritic process (Fig. 4a). In the contralateral side α-syn immunostaining was observed in the projecting zone in the inner layer of the molecular layer of the dentate (Fig. 4a). LV-α-syn DNA was only detected in the hippocampus of the side injected (ipsilateral) (Fig. 4b), but not the contralateral side in all three genotypes tested (Fig. 4b). In contrast, mice that received injection of LV-GFP showed signal only in neurons cells in the ipsilateral side, but little or no GFP signal was observed in axons or the contra-lateral side (Fig. 4c). By PCR, the GFP DNA was detected in the ipsilateral side but not in the contralateral (Fig. 4d). For both, the α-syn and GFP levels of DNA in the contra-lateral side were comparable to background.

**Fig. 3:** Confocal image analysis of α-syn localization in the contralateral side in α-syn KO, non-tg, and α-syn tg mice. Brain sections were immunolabeled with antibodies against CT-truncated α-syn and phosphorylated neurofilaments (p-NF; axonal marker). **a** Confocal image analysis of α-syn (red) and p-NF(green) in the (**a**) hippocampus and (**b**) axonal tracts on the contralateral side in α-syn KO, non-tg, and α-syn tg mice. White arrowhead indicates landmark for each image set. Scale bar = 10 μm. *N* = 5 per group

**Fig. 4:** Immunofluorescent and PCR analysis of LV-DNA in the hippocampus of α-syn KO, non-tg and α-syn tg mice. **a** Representative immunofluorescent images with an anti-synuclein antibody (syn-211) at low and high magnification of the contra- and ipsi-lateral CA1 hippocampal regions following unilateral LV-α-syn injection. In the ipsilateral side α-syn was detected in nerve cell bodies and neurites in the hippocampus, and in the contralateral side in the molecular layer of the dentate gyrus. **b** By PCR LV-α-syn was detected at high levels in the ipsilateral side and at background levels in the contralateral side. **c** Representative fluorescent images at low and high magnification of the contra- and ipsi-lateral CA1 hippocampal regions following unilateral LV-GFP injection. GFP was detected primarily in the neuronal cell bodies in the ipsilateral but not in the contralateral side. **d** LV-GFP DNA was detectable above background levels in the ipsilateral but not the contralateral side in all genotypes. For all experiments, PCR expression of LV DNA was normalized to GAPDH. *P <0.05 using a Student’s *t*-test comparing contra- and ipsilateral sides within a genotype. *N* = 5 per group. Low magnification scale bar = 100 μm; high magnification scale bar = 10 μm

The article "Anti-α-synuclein immunotherapy reduces α-synuclein propagation in the axon and degeneration in a combined viral vector and transgenic model of synucleinopathy" was retracted in 2026. Reasons: duplicated images; overlap with earlier publications; unreliable data.

### Passive immunotherapy reduces α-syn axonal accumulation and transport to the contra-lateral side following unilateral LV-α-syn injection

First, to confirm that the antibody trafficked into the CNS, Alexa-tagged 27-1 or 1H7 were injected into the tail vein and the brains analyzed 24 h after the injection. While with the 27-1 control, little or no fluorescent signal was detected in the CNS, in α-syn KO, non-tg and α-syn tg mice that received LV-α-syn injections, fluorescent Alexa signal was detected associated with neurons in a granular fashion (Fig. 5). To assess the effects of immunotherapy in the axonal transport and accumulation, groups of LV-α-syn-injected α-syn-KO, non-tg and α-syn tg mice were immunized weekly with intraperitoneal injections (30 mg/Kg) of either control IgG (27-1) or the 1H7 antibody (Fig. 1c) for a total 13 weeks, starting 1 week post-LV injection (Fig. 1a). Both the 1H7 antibody and 21-1 control immunotherapies were well-tolerated with all of the mice remaining healthy and with similar weight gains across groups. The α-syn-KO mice treated with 27-1 showed abundant expression and accumulation of α-syn in the hippocampus ipsilateral to the injection while in the contralateral side, α-syn was present in axons and in the molecular layer of the dentate gyrus (Fig. 6a, b). In contrast in animals treated with the 1H7 antibody there was approximately a 45% reduction (*P* < 0.05) in α-syn both ipsi- and contra-lateral to the site of injection (Fig. 6a, b), when compared to the isotype control group.

The article "Anti-α-synuclein immunotherapy reduces α-synuclein propagation in the axon and degeneration in a combined viral vector and transgenic model of synucleinopathy" was retracted in 2026. Reasons: duplicated images; overlap with earlier publications; unreliable data.

**Fig. 5:** Confocal analysis of systemic antibody trafficking to the CNS. Representative images from α-Syn KO, non-tg, and α-syn tg mice that were systemically injected (tail vein) with either Alexa-tagged 27-1 (control) or 1H7 antibodies and the brains were analyzed 24 h later. *N* = 3. Scale bar = 15 μm

**Fig. 6:** Immunohistochemical analysis of passively immunized mice following unilateral LV-α-syn injection. α-Syn KO, non-tg, and α-syn tg mice were passively immunized weekly for 13 weeks with intraperitoneal injections of either 27-1 (control) or 1H7 (α-syn antibody) beginning one week after LV-α-syn unilateral injection. Pathological analysis was conducted 16 weeks following unilateral LV-α-syn injection. Photomicrographs are of low and high magnification, with the high magnification image identified by the boxed-inset in the low magnification images. For these experiments an antibody against total α-syn was used. **a** Representative photomicrographs and (**b**) computer-aided analysis of contra- and ipsi-lateral hippocampus immunostained with an antibody against α-syn from α-syn KO mice immunized with 27-1 (control; *n* = 8) or 1H7 (α-syn antibody; *n* = 9). **c** Representative photomicrographs and (**d**) computer-aided analysis of contra- and ipsi-lateral hippocampus immunostained with an antibody against α-syn from non-tg mice immunized with 27-1 (control; *n* = 8) or 1H7 (α-syn antibody; *n* = 9). **e** Representative photomicrographs and (**f**) computer-aided analysis of contra- and ipsi-lateral hippocampus immunostained with an antibody against α-syn from α-syn tg mice immunized with 27-1 (control; *n* = 8) or 1H7 (α-syn antibody; *n* = 8). *P-value < 0.05 using ANOVA followed by Dunnett’s post-hoc test comparing 27-1 (control) and 1H7 (antibody) within a hemisphere, and ^#^ *P*-value < 0.05 using ANOVA followed by Tukey-Kramer post ho test comparing contra- and ipsilateral sides. Low magnification scale bar = 100 μm. High magnification scale bar = 25 μm

Similarly, non-tg mice (Fig. 6c, d) and α-syn tg mice (Fig. 6e, f) treated with 27-1 showed increased expression and accumulation of α-syn in the hippocampus ipsilateral and contralateral to the injection when compared to non-injected mice. Both the non-tg and α-syn tg mice treated with the 1H7 antibody showed a significant (*p* < 0.05) and robust reduction in α-syn axonal accumulation and pathology in both the ipsilateral and contralateral sides compared to IgG control (Fig. 6c, d).

More detailed analysis of the axons along the ipsi- and contra-lateral sides showed accumulation of α-syn in the axons and in dystrophic neurites in the 27-1 treated α-syn KO (Fig. 7a), non-tg (Fig. 7b), and α-syn tg (Fig. 7c) animals, while the 1H7-treated mice presented substantially lower levels of axonal pathology in all three genotypes (Fig. 7a-c).

The article "Anti-α-synuclein immunotherapy reduces α-synuclein propagation in the axon and degeneration in a combined viral vector and transgenic model of synucleinopathy" was retracted in 2026. Reasons: duplicated images; overlap with earlier publications; unreliable data.

**Fig. 7:** Effects of passive immunization on axonal accumulation of α-syn in ipsi- and contralateral sides. α-Syn KO, non-tg, and α-syn tg mice were passively immunized (intraperitoneal injections) weekly for 13 weeks with either 27-1 (control) or 1H7 (α-syn antibody) beginning one week after LV-α-syn unilateral injection. Pathological analysis was conducted 16 weeks following unilateral LV-α-syn injection. Representative photomicrographs of total α-syn accumulation in hippocampal axons in (**a**) α-syn KO, (**b**) non-tg, and (**c**) α-syn tg mice. Arrows indicate dystrophic neurites. Scale bar = 25 μm

### Immunization with the 1H7 antibody reduces the α-syn mediated degeneration of axons following unilateral LV-α-syn injection

Next, we investigated the effects of the immunotherapy on the axonal pathology. For this purpose, sections were immunostained with the SMI312 antibody against phosphorylated neurofilaments and analyzed by confocal microscopy. Interestingly, both IgG treated α-syn-KO (Fig. 8a, b) and non-tg mice (Fig. 8c, d) displayed a significant (*p* < 0.05) reduction in axons immunostained with the SMI312 antibody in the contralateral side, when compared to the ipsilateral side, indicating that the axonal dissemination of α-syn might promote a higher degree of toxicity than the over-expression of that protein itself. When treated with 1H7 antibody, both α-syn KO (8A, B) and non-tg (8C, D) mice displayed significantly higher levels of intact SMI312 immunoreactive axons (*P* < 0.05) when compared to IgG control. A substantially higher degree of axonal loss was observed in α-syn tg mice in both ipsi- and contralateral sides of LV-α-syn injection, when compared to the other genotypes (Fig. 8e, f). Strikingly, despite this higher level of axonal pathology in α-syn tg mice, the immunization with 1H7 antibody significantly protected against the axonal loss in this genotype (*P* < 0.05 compared to 27-1) and to levels found in comparable other genotypes (Fig. 8b, d). In order to further investigate the relationship between the α-syn-associated axonal pathology and the effects of immunotherapy, brain sections were double labeled with antibodies against α-syn and the SMI312 antibody. Consistent with the results discussed above, mice of all three genotypes injected with LV-α-syn showed a higher degree of colocalization between α-syn and SMI312 in dystrophic neurites in the contralateral side of IgG control (27-1) versus 1H7-treated mice (Fig. 9a). Immunization with 1H7 antibody resulted in a significant reduction (*p* < 0.05) of 50%, 35% and 25% in α-syn/SMI312 immunoreactive dystrophic neurites in the contralateral side in the α-syn-KO, non-tg and α-syn tg mice, respectively (Fig. 9b, c). Taken together these results support the notion that the 1H7 antibody reduced the axonal transport and accumulation of α-syn and prevented the associated axonal pathology, irrespective of the baseline levels of α-syn expression.

The article "Anti-α-synuclein immunotherapy reduces α-synuclein propagation in the axon and degeneration in a combined viral vector and transgenic model of synucleinopathy" was retracted in 2026. Reasons: duplicated images; overlap with earlier publications; unreliable data.

**Fig. 8:** Confocal analysis of phosphorylated neurofilaments in 1H7 passively immunized mice. α-Syn KO, non-tg, and α-syn tg mice were passively immunized weekly for 13 weeks with either 27-1 (control) or 1H7 (α-syn antibody) beginning one week after LV-α-syn unilateral injection. Pathological analysis of axonal density using SMI312 antibody against phosphorylated neurofilaments was conducted 16 weeks following unilateral LV-α-syn injection. **a** Representative images and (**b**) computer-aided analysis of axonal density in the contra- and ipsilateral side of α-syn KO mice. **c** Representative images and (**d**) computer-aided analysis of axonal density in the contra- and ipsilateral side of non-tg mice. **e** Representative images and (**f**) computer-aided analysis of axonal density in the contra- and ipsilateral side of α-syn tg mice. *P-value < 0.05 using ANOVA followed by Dunnett’s post-hoc test comparing 27-1 (control) and 1H7 (antibody) within a hemisphere. ^#^ *P* < 0.05 using ANOVA followed by Tukey-Kramer post hoc test comparing contra- and ipsilateral sides. Scale bar = 30 μm

**Fig. 9:** Co-localization of neurofilament marker SMI312 and CT-α-syn was reduced in passively immunized α-syn tg mice. To analyze if passive immunization altered the subcellular distribution of CT-α-syn, double labeling of brain sections of α-syn KO, non-tg, and α-syn tg mice that were passively immunized weekly for 13 weeks with either 27-1 (control) or 1H7 (α-syn antibody) beginning one week after LV-α-syn unilateral injection were analyzed using SMI312 antibody against phosphorylated neurofilaments (p-NF) and the CT-α-syn antibody SYN105 was conducted 14 weeks following unilateral LV-α-syn injection. **a** Representative confocal images of the contralateral neuropil in brain sections from α-syn KO, non-tg, and α-syn tg mice immunized with 27-1 (control), or (**b**) immunized with 1H7 (antibody). Arrows indicate co-localization of the SMI312 signal with CT-α-syn in neurofilament-like structures. **c** Analysis of the percentage of co-localization between the neurofilament marker SMI312 and the CT-α-syn antibody SYN105. Error bars represent ± SEM. *P <0.05 when statistically analyzed using a Student’s *t*-test. Scale bar = 25 μm. α-Syn KO mice + 27-1 (control) *n* = 8; α-syn KO + 1H7 antibody *n* = 9; non-tg mice + 27-1 (control) *n* = 10; non-tg mice + 1H7 antibody *n* = 9; α-syn tg mice + 27-1 (control) *n* = 8; α-syn tg mice + 1H7 antibody *n* = 8

To determine if in the immunized mice, microglial clearance plays a role in the removal of propagating α-syn, double-labeling studies were performed in sections of the α-syn KO, non-tg and α-syn tg mice injected with LV-α-syn and treated with 27-1 (control) or 1H7 antibody (Fig. 10). In mice treated with 27-1, microglia (FITC, green channel)) was detected in the proximity to small granular aggregates of α-syn (Tyramide red, red channel) but little (under 1%) (Fig. 10c). In contrast, mice treated with 1H7 showed a higher proportion of microglia containing granular deposits of α-syn (Fig. 10b and c).

The article "Anti-α-synuclein immunotherapy reduces α-synuclein propagation in the axon and degeneration in a combined viral vector and transgenic model of synucleinopathy" was retracted in 2026. Reasons: duplicated images; overlap with earlier publications; unreliable data.

**Fig. 10:** Co-localization of microglial marker Iba-1 and α-syn was increased in passively immunized α-syn tg mice. To analyze if passive immunization was associated with microglial clearance of α-syn, double labeling of brain sections of α-syn KO, non-tg, and α-syn tg mice that were passively immunized weekly for 13 weeks with either 27-1 (control) or 1H7 (α-syn antibody) beginning one week after LV-α-syn unilateral injection were analyzed using Iba-1 antibody against microglia and α-syn (syn-211)-positive aggregates was conducted 14 weeks following unilateral LV-α-syn injection. Double labeled sections were analyzed with the laser scanning confocal microscope. Panels in red represents α-syn (syn-211 antibody), and green represents Iba-1(**a**) Representative confocal images of the contralateral hippocampal neuropil in brain sections from α-syn KO, non-tg, and α-syn tg mice immunized with 27-1 (control), or (**b**) immunized with 1H7 (antibody). Arrows indicate co-localization of the Iba-1 signal with α-syn in microglia. **c** Analysis of the percentage of co-localization between the microglial marker Iba-1 and the α-syn syn-211 antibody. Error bars represent ± SEM. α-Syn KO mice + 27-1 (control) *n* = 8; α-syn KO + 1H7 antibody *n* = 9; non-tg mice + 27-1 (control) *n* = 10; non-tg mice + 1H7 antibody *n* = 9; α-syn tg mice + 27-1 (control) *n* = 8; α-syn tg mice + 1H7 antibody *n* = 8. Scale bar = 10 μm

### Effects of passive immunization with the 1H7 antibody in the water maze task in a viral vector model of α-syn mediated axonal pathology

In order to evaluate the effects of passive immunization with the α-syn antibody on memory and learning in the combined tg and lentivirus model, groups of α-syn-KO, non-tg and α-syn tg mice that received unilateral intra-hippocampal LV-α-syn injection were tested in the water maze following the immunization period (13 weeks) (Fig. 1a). During the initial training part of the test when the platform was visible (cued; days 1-3), all groups performed at comparable levels as determined by repeated measures two-way ANOVA (Fig. 11a).

The article "Anti-α-synuclein immunotherapy reduces α-synuclein propagation in the axon and degeneration in a combined viral vector and transgenic model of synucleinopathy" was retracted in 2026. Reasons: duplicated images; overlap with earlier publications; unreliable data.

**Fig. 11:** Passive immunization with CT-α-syn antibodies improved behavioral deficits in α-syn KO and α-syn tg mice. The effect of immunization with CT**-**α syn antibodies on learning as well as memory and motor performance were analyzed by water maze. **a** Performance in the water maze (distance to the platform) during the cued with submerged platform tests in mice immunized with 27-1 (control), or with 1H7 (antibody). **b** Probe test performance, measured as the time spent in correct quadrant by mice passively immunized with either 27-1 or 1H7 antibodies. Error bars represent ± SEM. *P < 0.05 when comparing 27-1-immunized mice to 1H7-immunized mice within genotype. α-Syn KO mice + 27-1 (control) *n* = 8; α-syn KO + 1H7 antibody *n* = 9; non-tg mice + 27-1 (control) *n* = 10; non-tg mice + 1H7 antibody *n* = 9; α-syn tg mice + 27-1 (control) *n* = 8; α-syn tg mice + 1H7 antibody *n* = 8

Following the cued platform session, the mice underwent 4 days of testing during which the platform was submerged and hidden from view (days 4-7). On the first day of testing with the hidden platform the non-tg and α-syn tg performed comparably, however the α-syn KO mice displayed some deficits (Fig. 11a). Over the next 3 days of testing, the performance of both the 27-1- and 1H7-treated non-tg mice improved in terms of the distance of their swim path and the time taken to locate the platform (Fig. 11a). In contrast, the performance of the 27-1-treated α-syn tg mice did not improve to the same extent (Fig. 9a) and a significant difference was observed between the 27-1-treated α-syn tg mice and non-tg mice. The α-syn tg mice immunized with the 1H7 took a significantly shorter time to locate the hidden platform in comparison to 27-1-treated α-syn tg mice (Fig. 11a) indicating that passive immunization with those antibodies was able to ameliorate the memory and learning deficits observed in the 27-1-treated α-syn tg mice. In contrast, both the 27-1 and 1H7 treated α-syn KO mice required more time to find the submerged platform (Fig. 11a).

On day 8, the platform was removed and time expended in the quadrant where the platform was located was analyzed (probe test). The α-syn KO mice treated with 27-1 expended less time in the target quadrant while mice treated with 1H7 displayed a trend toward more time in the target quadrant (Fig. 11b). For the non-tg mice both the 27-1 and 1H7 treated mice remained most of the recorded time in the target quadrant (Fig. 11b). Finally, the 27-1 treated α-syn tg mice expended less time in the target quadrant while α-syn tg treated with 1H7 expended more time comparable with the non-tg mice (Fig. 11b).

The article "Anti-α-synuclein immunotherapy reduces α-synuclein propagation in the axon and degeneration in a combined viral vector and transgenic model of synucleinopathy" was retracted in 2026. Reasons: duplicated images; overlap with earlier publications; unreliable data.

## Discussion

The present study developed a new mouse model of dissemination and accumulation of α-syn in axons on the contralateral side by performing unilateral intra-cerebral injections with a LV-α-syn vector construct in non-tg, α-syn KO, and α-syn tg mice. We then used this model to assess the effects of passive immunization with the anti-α-syn antibody 1H7 on the axonal transport and accumulation of α-syn in α-syn KO, non-tg and α-syn tg mice that received unilateral intra-hippocampal injection with a lentivirus expressing human α-syn. Previous studies have shown that α-syn oligomers can be released by affected neurons and transmit trans-axonally and through other mechanisms such as release of free α-syn, exoxomes or nanotubules to adjacent neurons and glial cells leading to neurotoxicity and inflammatory responses [2, 3, 8, 10, 12, 31, 35], thus suggesting that immunotherapy might prevent pathological responses by neutralizing α-syn species and blocking transmission [72].

Using the approach of unilaterally injecting LV-α-syn in the hippocampus, we were able to observe axonal transport and accumulation of α-syn in the contra-lateral hemisphere. One likely mechanism for the accumulation of α-syn in the contra-lateral hemisphere is trans-synaptic propagation [30] in which α-syn is transmitted from the pre-synaptic neuron originating in the ipsi-lateral hemisphere to post-synaptic neuron in the contra-lateral hemisphere. Our results are consistent with previous studies that injected pre-formed α-syn fibrils into the olfactory bulb [38], striatum [38] or adeno-associated viral vector (AAV)-α-syn into the vagus nucleus [71]. These models of α-syn propagation used wt mice, which were injected unilaterally, and the α-syn propagation was followed sequentially through various connected brain regions, as well as in the contralateral brain region [54]. While preformed α-syn fibrils have a limiting half-life, viral vector models continuously expressing α-syn can overcome this limitation allowing for the long-term study of α-syn [54]. Consistent with these previous studies, the present study showed abnormal patterns of α-syn accumulations along axons, often associated with axonal dystrophy, as well as accumulation of the protein in neuronal bodies of contralateral hippocampus. While the presence of α-syn in axons could be explained by transport of α-syn along the commissural fibers that interconnect both hippocampi, the presence of intra-somatic α-syn pathology is suggestive of trans-synaptic propagation, and expands upon these previous models, which evaluated α-syn propagation from the olfactory bulb [38] and brain stem [71], respectively.

The article "Anti-α-synuclein immunotherapy reduces α-synuclein propagation in the axon and degeneration in a combined viral vector and transgenic model of synucleinopathy" was retracted in 2026. Reasons: duplicated images; overlap with earlier publications; unreliable data.

Unlike previous papers using tg or viral vector to study local immunization against α-syn, we demonstrated the effects of an α-syn monoclonal antibody, 1H7, administered systemically using the LV-α-syn model. Anti-α-syn immunizations have been previously shown to be effective in AAV-α-syn propagation models using N-terminal α-syn antibody by blocking α-syn accumulation [71]. 1H7 was previously demonstrated to reduce the accumulation and propagation of CT-truncated α-syn and improved axonal and motor deficits via a mechanism that might involve protecting α-syn from CT cleavage in the extracellular space in a transgenic α-syn mouse model [19].

Both in the current study and in previous study [19] we showed that 1H7 was effective *in vivo*. While the mechanism of action for how 1H7 immunization blocked α-syn propagation has yet to be determined, it is possible the antibody bound and neutralized extracellular α-syn species, preventing their binding to neurons and internalization into the cytoplasm [3]. Furthermore, once opsonized by the 1H7 antibody, the α-syn aggregates may be cleared by microglial phagocytosis [34], which has also been suggested as the major scavenger of extracellular α-syn. Supporting this hypothesis is our current finding that microglia co-localized with α-syn, which is indicative of extracelluar α-syn clearance by microglia in a similar manner to what has been previously reported [34], It is also possible that the 1H7 antibody works by blocking binding to and uptake by neurons, halting templating and neuron-to-neuron propagation [66]. An alternate mechanism for 1H7 includes the possible inhibition of α-syn aggregation. Since 1H7 binds to an epitope proximal to the non-amyloid β component (NAC) region of a-syn, the antibody might potentially mask hydrophobic pockets and modify α-syn folding states that are required for self aggregation.

We also show that immunotherapy in our model of α-syn axonal transport and accumulation improved axonal pathology. Dickson et al. has previously described extensive hippocampal pathology in Lewy body disease [15]. In our LV-α-syn models we recapitulated the hippocampal pathology and then applied immunotherapy to mitigate the axonal pathology and improved synaptic trafficking and axonal transport, although it is possible that the antibody has additional mechanisms further downstream which partially contribute to reduced α-syn.

The article "Anti-α-synuclein immunotherapy reduces α-synuclein propagation in the axon and degeneration in a combined viral vector and transgenic model of synucleinopathy" was retracted in 2026. Reasons: duplicated images; overlap with earlier publications; unreliable data.

## Conclusions

Here we developed a new model of α-syn transmission in mice to test the effects of anti-α-syn antibodies at decreasing synuclein trans-axonal dissemination and related deficits. We show that a new antibody, denominated 1H7, that recognizes α-syn 91-99 aa residues was effective at mitigating the axonal pathology and improved synaptic trafficking and axonal transport, although it is possible that the antibody has additional mechanisms further downstream which partially contribute to reduced α-syn. Together this study supports the notion that passive immunotherapy with antibodies targeting specific domains of α-syn are capable of reducing axonal transport and accumulation of α-syn from ipsi-lateral to contra-lateral hemispheres and provides a novel mechanism trough which immunotherpay might be of potential interest to the treatment of PD, DLB and related synucleinopathies.

## Abbreviations

AAV: Adeno-associated viral vector
Ab: Antibody
CT: C-terminal
Ct: Threshold cycle
DLB: Dementia with Lewy bodies
ELISA: Enzyme-linked immunosorbent assay
KO: Knock out
LSCM: Laser scanning confocal microscope
LV: Lentivirus
NAC: Non-amyloid β component
PD: Parkinson’s disease
PDD: Parkinson’s disease dementia
Tg: Transgenic
UCSD: University of California San Diego
α-syn: α-synuclein

## References

[1] Abeliovich A, Schmitz Y, Farinas I, Choi-Lundberg D, Ho WH, Castillo PE, Shinsky N, Verdugo JM, Armanini M, Ryan A (2000). Mice lacking alpha-synuclein display functional deficits in the nigrostriatal dopamine system. Neuron.

[2] Angot E, Steiner JA, Lema Tome CM, Ekstrom P, Mattsson B, Bjorklund A, Brundin P (2012). Alpha-synuclein cell-to-cell transfer and seeding in grafted dopaminergic neurons in vivo. PLoS One.

[3] Bae EJ, Lee HJ, Rockenstein E, Ho DH, Park EB, Yang NY, Desplats P, Masliah E, Lee SJ (2012). Antibody-aided clearance of extracellular alpha-synuclein prevents cell-to-cell aggregate transmission. J Neurosci.

[4] Bar-On P, Crews L, Koob AO, Mizuno H, Adame A, Spencer B, Masliah E (2008). Statins reduce neuronal alpha-synuclein aggregation in in vitro models of Parkinson’s disease. J Neurochem.

[5] Bellucci A, Zaltieri M, Navarria L, Grigoletto J, Missale C, Spano P (2012). From alpha-synuclein to synaptic dysfunctions: new insights into the pathophysiology of Parkinson’s disease. Brain Res.

[6] Braak H, Braak E (2000). Pathoanatomy of Parkinson’s disease. J Neurol.

[7] Braak H, Brettschneider J, Ludolph AC, Lee VM, Trojanowski JQ, Del Tredici K (2013). Amyotrophic lateral sclerosis--a model of corticofugal axonal spread. Nat Rev Neurol.

[8] Brundin P, Melki R, Kopito R (2010). Prion-like transmission of protein aggregates in neurodegenerative diseases. Nat Rev Mol Cell Biol.

The article "Anti-α-synuclein immunotherapy reduces α-synuclein propagation in the axon and degeneration in a combined viral vector and transgenic model of synucleinopathy" was retracted in 2026. Reasons: duplicated images; overlap with earlier publications; unreliable data.

[9] Conway KA, Harper JD, Lansbury PT (1998). Accelerated in vitro fibril formation by a mutant alpha-synuclein linked to early-onset Parkinson disease. Nat Med.

[10] Danzer KM, Kranich LR, Ruf WP, Cagsal-Getkin O, Winslow AR, Zhu L, Vanderburg CR, McLean PJ (2012). Exosomal cell-to-cell transmission of alpha synuclein oligomers. Mol Neurodegener.

[11] Danzer KM, Ruf WP, Putcha P, Joyner D, Hashimoto T, Glabe C, Hyman BT, McLean PJ (2011). Heat-shock protein 70 modulates toxic extracellular alpha-synuclein oligomers and rescues trans-synaptic toxicity. FASEB J.

[12] Desplats P, Lee HJ, Bae EJ, Patrick C, Rockenstein E, Crews L, Spencer B, Masliah E, Lee SJ (2009). Inclusion formation and neuronal cell death through neuron-to-neuron transmission of alpha-synuclein. Proc Natl Acad Sci U S A.

[13] Dickson DW (2001). Alpha-synuclein and the Lewy body disorders. Curr Opin Neurol.

[14] Dickson D, Lin W-L, Liu W-K, Yen S-H (1999). Multiple system atrophy: a sporadic synucleinopathy. Brain Pathol.

[15] Dickson DW, Schmidt ML, Lee VM, Zhao ML, Yen SH, Trojanowski JQ (1994). Immunoreactivity profile of hippocampal CA2/3 neurites in diffuse Lewy body disease. Acta Neuropathol (Berl).

[16] Fleming SM, Salcedo J, Fernagut PO, Rockenstein E, Masliah E, Levine MS, Chesselet MF (2004). Early and progressive sensorimotor anomalies in mice overexpressing wild-type human alpha-synuclein. J Neurosci.

[17] Franklin KBJ, Paxinos G (1997). The mouse brain in stereotaxic coordinates.

[18] Games D, Seubert P, Rockenstein E, Patrick C, Trejo M, Ubhi K, Ettle B, Ghassemiam M, Barbour R, Schenk D (2013). Axonopathy in an alpha-synuclein transgenic model of Lewy body disease is associated with extensive accumulation of C-terminal-truncated alpha-synuclein. Am J Pathol.

[19] Games D, Valera E, Spencer B, Rockenstein E, Mante M, Adame A, Patrick C, Ubhi K, Nuber S, Sacayon P (2014). Reducing C-terminal-truncated alpha-synuclein by immunotherapy attenuates neurodegeneration and propagation in Parkinson’s disease-like models. J Neurosci.

[20] Hansen C, Angot E, Bergstrom AL, Steiner JA, Pieri L, Paul G, Outeiro TF, Melki R, Kallunki P, Fog K (2011). Alpha-Synuclein propagates from mouse brain to grafted dopaminergic neurons and seeds aggregation in cultured human cells. J Clin Invest.

[21] Hashimoto M, Masliah E (1999). Alpha-synuclein in Lewy body disease and Alzheimer’s disease. Brain Pathol.

[22] Helwig M, Klinkenberg M, Rusconi R, Musgrove RE, Majbour NK, El-Agnaf OM, Ulusoy A, Di Monte DA (2016). Brain propagation of transduced alpha-synuclein involves non-fibrillar protein species and is enhanced in alpha-synuclein null mice. Brain.

The article "Anti-α-synuclein immunotherapy reduces α-synuclein propagation in the axon and degeneration in a combined viral vector and transgenic model of synucleinopathy" was retracted in 2026. Reasons: duplicated images; overlap with earlier publications; unreliable data.

[23] Iwai A (2000). Properties of NACP/alpha-synuclein and its role in Alzheimer’s disease. Biochim Biophys Acta.

[24] Iwai A, Yoshimoto M, Masliah E, Saitoh T (1995). Non-A beta component of Alzheimer’s disease amyloid (NAC) is amyloidogenic. Biochemistry.

[25] Iwatsubo T, Yamaguchi H, Fujimuro M, Yokosawa H, Ihara Y, Trojanowski JQ, Lee V-M (1996). Purification and characterization of Lewy bodies from brains of patients with diffuse Lewy body disease. AmJPathol.

[26] Jones DR, Delenclos M, Baine AT, DeTure M, Murray ME, Dickson DW, McLean PJ (2015). Transmission of soluble and insoluble alpha-synuclein to mice. J Neuropath Exp Neurol.

[27] Kim C, Ho DH, Suk JE, You S, Michael S, Kang J, Joong Lee S, Masliah E, Hwang D, Lee HJ (2013). Neuron-released oligomeric alpha-synuclein is an endogenous agonist of TLR2 for paracrine activation of microglia. Nat Commun.

[28] Kramer ML, Schulz-Schaeffer WJ (2007). Presynaptic alpha-synuclein aggregates, not Lewy bodies, cause neurodegeneration in dementia with Lewy bodies. J Neurosci.

[29] Lansbury PT (1999). Evolution of amyloid: what normal protein folding may tell us about fibrillogenesis and disease. Proc Natl Acad Sci U S A.

[30] Lashuel HA, Overk CR, Oueslati A, Masliah E (2013). The many faces of alpha-synuclein: from structure and toxicity to therapeutic target. Nat Rev Neurosci.

[31] Lee SJ, Desplats P, Lee HJ, Spencer B, Masliah E (2012). Cell-to-cell transmission of alpha-synuclein aggregates. Methods Mol Biol.

[32] Lee SJ, Desplats P, Sigurdson C, Tsigelny I, Masliah E (2010). Cell-to-cell transmission of non-prion protein aggregates. Nat Rev Neurol.

[33] Lee HJ, Suk JE, Bae EJ, Lee JH, Paik SR, Lee SJ (2008) Assembly-dependent endocytosis and clearance of extracellular alpha-synuclein. Int J Biochem Cell Biol 40(9):1835-49.10.1016/j.biocel.2008.01.01718291704

[34] Lee HJ, Suk JE, Bae EJ, Lee SJ (2008). Clearance and deposition of extracellular alpha-synuclein aggregates in microglia. Biochem Biophys Res Commun.

[35] Lee HJ, Suk JE, Patrick C, Bae EJ, Cho JH, Rho S, Hwang D, Masliah E, Lee SJ (2010). Direct transfer of alpha-synuclein from neuron to astroglia causes inflammatory responses in synucleinopathies. J Biol Chem.

[36] Loov C, Scherzer CR, Hyman BT, Breakefield XO, Ingelsson M (2016). Alpha-synuclein in extracellular vesicles: functional implications and diagnostic opportunities. Cell Mol Neurobiol.

[37] Luk KC, Kehm V, Carroll J, Zhang B, O'Brien P, Trojanowski JQ, Lee VM (2012). Pathological alpha-synuclein transmission initiates Parkinson-like neurodegeneration in nontransgenic mice. Science.

[38] Luk KC, Kehm VM, Zhang B, O'Brien P, Trojanowski JQ, Lee VM (2012). Intracerebral inoculation of pathological alpha-synuclein initiates a rapidly progressive neurodegenerative alpha-synucleinopathy in mice. J Exp Med.

The article "Anti-α-synuclein immunotherapy reduces α-synuclein propagation in the axon and degeneration in a combined viral vector and transgenic model of synucleinopathy" was retracted in 2026. Reasons: duplicated images; overlap with earlier publications; unreliable data.

[39] Mandler M, Valera E, Rockenstein E, Mante M, Weninger H, Patrick C, Adame A, Schmidhuber S, Santic R, Schneeberger A (2015). Active immunization against alpha-synuclein ameliorates the degenerative pathology and prevents demyelination in a model of multiple system atrophy. Mol Neurodegener.

[40] Marr RA, Rockenstein E, Mukherjee A, Kindy MS, Hersh LB, Gage FH, Verma IM, Masliah E (2003). Neprilysin gene transfer reduces human amyloid pathology in transgenic mice. J Neurosci.

[41] Marxreiter F, Ettle B, May VE, Esmer H, Patrick C, Kragh CL, Klucken J, Winner B, Riess O, Winkler J (2013). Glial A30P alpha-synuclein pathology segregates neurogenesis from anxiety-related behavior in conditional transgenic mice. Neurobiol Dis.

[42] Masliah E, Mallory M, Hansen L, Alford M, DeTeresa R, Terry R (1993). An antibody against phosphorylated neurofilaments identifies a subset of damaged association axons in Alzheimer’s disease. AmJPathol.

[43] Masliah E, Rockenstein E, Adame A, Alford M, Crews L, Hashimoto M, Seubert P, Lee M, Goldstein J, Chilcote T (2005). Effects of alpha-synuclein immunization in a mouse model of Parkinson’s disease. Neuron.

[44] Masliah E, Rockenstein E, Mante M, Crews L, Spencer B, Adame A, Patrick C, Trejo M, Ubhi K, Rohn TT (2011). Passive immunization reduces behavioral and neuropathological deficits in an alpha-synuclein transgenic model of Lewy body disease. PLoS One.

[45] Masliah E, Rockenstein E, Veinbergs I, Mallory M, Hashimoto M, Takeda A, Sagara Y, Sisk A, Mucke L (2000). Dopaminergic loss and inclusion body formation in alpha-synuclein mice: implications for neurodegenerative disorders. Science.

[46] Masliah E, Rockenstein E, Veinbergs I, Sagara Y, Mallory M, Hashimoto M, Mucke L (2001). beta-amyloid peptides enhance alpha-synuclein accumulation and neuronal deficits in a transgenic mouse model linking Alzheimer’s disease and Parkinson’s disease. Proc Natl Acad Sci U S A.

[47] Mason DM, Nouraei N, Pant DB, Miner KM, Hutchison DF, Luk KC, Stolz JF, Leak RK (2016). Transmission of alpha-synucleinopathy from olfactory structures deep into the temporal lobe. Mol Neurodegener.

[48] McKeith IG (2000). Spectrum of Parkinson’s disease, Parkinson’s dementia, and Lewy body dementia. Neurol Clin.

[49] NIA (2015) Lewy Body Dementia: Information for Patients, Families, and Professionals., https://www.nia.nih.gov/alzheimers/publication/lewy-body-dementia/basics-lewy-body-dementia. Accessed 3 Jan 2017.

[50] Olanow CW, Brundin P (2013). Parkinson’s disease and alpha synuclein: is Parkinson’s disease a prion-like disorder?. Mov Disord.

The article "Anti-α-synuclein immunotherapy reduces α-synuclein propagation in the axon and degeneration in a combined viral vector and transgenic model of synucleinopathy" was retracted in 2026. Reasons: duplicated images; overlap with earlier publications; unreliable data.

[51] Oueslati A, Fournier M, Lashuel HA (2010). Role of post-translational modifications in modulating the structure, function and toxicity of alpha-synuclein: implications for Parkinson’s disease pathogenesis and therapies. Prog Brain Res.

[52] Peelaerts W, Bousset L, Van der Perren A, Moskalyuk A, Pulizzi R, Giugliano M, Van den Haute C, Melki R, Baekelandt V (2015). Alpha-Synuclein strains cause distinct synucleinopathies after local and systemic administration. Nature.

[53] Prusiner SB, Woerman AL, Mordes DA, Watts JC, Rampersaud R, Berry DB, Patel S, Oehler A, Lowe JK, Kravitz SN (2015). Evidence for alpha-synuclein prions causing multiple system atrophy in humans with parkinsonism. Proc Natl Acad Sci U S A.

[54] Rey NL, George S, Brundin P (2016). Review: Spreading the word: precise animal models and validated methods are vital when evaluating prion-like behaviour of alpha-synuclein. Neuropathol Appl Neurobiol.

[55] Rey NL, Petit GH, Bousset L, Melki R, Brundin P (2013). Transfer of human alpha-synuclein from the olfactory bulb to interconnected brain regions in mice. Acta Neuropathol.

[56] Rey NL, Steiner JA, Maroof N, Luk KC, Madaj Z, Trojanowski JQ, Lee VM, Brundin P (2016). Widespread transneuronal propagation of alpha-synucleinopathy triggered in olfactory bulb mimics prodromal Parkinson’s disease. J Exp Med.

[57] Rockenstein E, Mallory M, Hashimoto M, Song D, Shults CW, Lang I, Masliah E (2002). Differential neuropathological alterations in transgenic mice expressing alpha-synuclein from the platelet-derived growth factor and Thy-1 promoters. J Neurosci Res.

[58] Roy S, Winton MJ, Black MM, Trojanowski JQ, Lee VM (2007). Rapid and intermittent cotransport of slow component-b proteins. J Neurosci.

[59] Savica R, Grossardt BR, Bower JH, Boeve BF, Ahlskog JE, Rocca WA (2013). Incidence of dementia with Lewy bodies and Parkinson disease dementia. JAMA Neurol.

[60] Spencer B, Potkar R, Trejo M, Rockenstein E, Patrick C, Gindi R, Adame A, Wyss-Coray T, Masliah E (2009). Beclin 1 gene transfer activates autophagy and ameliorates the neurodegenerative pathology in alpha-synuclein models of Parkinson’s and Lewy body diseases. J Neurosci.

[61] Spillantini MG, Schmidt ML, Lee VM, Trojanowski JQ, Jakes R, Goedert M (1997). Alpha-synuclein in Lewy bodies. Nature.

[62] Steiner JA, Angot E, Brundin P (2011). A deadly spread: cellular mechanisms of alpha-synuclein transfer. Cell Death Differ.

[63] Taschenberger G, Garrido M, Tereshchenko Y, Bahr M, Zweckstetter M, Kugler S (2012). Aggregation of alphaSynuclein promotes progressive in vivo neurotoxicity in adult rat dopaminergic neurons. Acta Neuropathol.

The article "Anti-α-synuclein immunotherapy reduces α-synuclein propagation in the axon and degeneration in a combined viral vector and transgenic model of synucleinopathy" was retracted in 2026. Reasons: duplicated images; overlap with earlier publications; unreliable data.

[64] Tiscornia G, Singer O, Verma IM (2006). Design and cloning of lentiviral vectors expressing small interfering RNAs. Nat Protoc.

[65] Toledo JB, Gopal P, Raible K, Irwin DJ, Brettschneider J, Sedor S, Waits K, Boluda S, Grossman M, Van Deerlin VM (2016). Pathological alpha-synuclein distribution in subjects with coincident Alzheimer’s and Lewy body pathology. Acta Neuropathol.

[66] Tran HT, Chung CH, Iba M, Zhang B, Trojanowski JQ, Luk KC, Lee VM (2014). Alpha-synuclein immunotherapy blocks uptake and templated propagation of misfolded alpha-synuclein and neurodegeneration. Cell Rep.

[67] Trojanowski J, Goedert M, Iwatsubo T, Lee V (1998). Fatal attractions: abnormal protein aggregation and neuron death in Parkinson’s disease and lewy body dementia. Cell Death Differ.

[68] Tsigelny IF, Sharikov Y, Miller MA, Masliah E (2008). Mechanism of alpha-synuclein oligomerization and membrane interaction: theoretical approach to unstructured proteins studies. Nanomedicine.

[69] Tyson T, Steiner JA, Brundin P (2015). Sorting out release, uptake and processing of alpha-synuclein during prion-like spread of pathology. J Neurochem.

[70] Ueda K, Fukushima H, Masliah E, Xia Y, Iwai A, Yoshimoto M, Otero DA, Kondo J, Ihara Y, Saitoh T (1993). Molecular cloning of cDNA encoding an unrecognized component of amyloid in Alzheimer disease. Proc Natl Acad Sci U S A.

[71] Ulusoy A, Rusconi R, Perez-Revuelta BI, Musgrove RE, Helwig M, Winzen-Reichert B, Di Monte DA (2013). Caudo-rostral brain spreading of alpha-synuclein through vagal connections. EMBO Mol Med.

[72] Valera E, Masliah E (2013). Immunotherapy for neurodegenerative diseases: Focus on alpha-synucleinopathies. Pharmacol Ther.

[73] Winner B, Jappelli R, Maji SK, Desplats PA, Boyer L, Aigner S, Hetzer C, Loher T, Vilar M, Campioni S (2011). In vivo demonstration that alpha-synuclein oligomers are toxic. Proc Natl Acad Sci U S A.

